# Association between Glucocorticoids and Mortality in Patients with Severe Pneumonia: A Systematic Review and Meta-Analysis Based on Randomized Controlled Trials

**DOI:** 10.1155/2022/1191205

**Published:** 2022-08-08

**Authors:** Qiufeng Tang, Qiongyan Chen, Yanqing Li, Zuanjin Wang

**Affiliations:** ^1^Department of Pharmacy, Geriatric Hospital of Hainan, Haikou, 571100 Hainan, China; ^2^Department of Respiratory Medicine, Danzhou People's Hospital, Danzhou, 571700 Hainan, China; ^3^Department of Emergency, 928th Hospital of PLA Joint Logistics Support Force, Haikou, 570216 Hainan, China

## Abstract

**Objective:**

To explore the associations between glucocorticoid use and the clinical outcome of patients with severe pneumonia.

**Methods:**

Medical databases including PubMed, EMBASE, and ScienceDirect were searched for relevant literature. Two independent researchers extracted the primary endpoint from the included literature. The Cochrane *Q* test and *I*^2^ statistics were used to evaluate the interstudy heterogeneity. The combined risk estimates were calculated by random effect model, and the source of heterogeneity was evaluated by subgroup analysis. Funnel plot and Egger's test were used to assess publication bias. *P* < 0.05 denoted statistical significance.

**Results:**

A total of 12 literature, including 8171 patients with 1083 deaths, were included in this study for meta-analysis. The use of glucocorticoids significantly increased the mortality (RR = 1.44, 95% CI: 1.13, 1.84, *P* < 0.001), the risk of requiring mechanical ventilation (RR = 1.62, 95% CI: 1.30, 2.02, *P* < 0.001), and the incidence of nosocomial infection (RR = 1.36, 95% CI: 1.01, 1.82, *P* = 0.04) in patients with severe pneumonia as compared with the control group. In addition, the use of glucocorticoids did not seem to be associated with length of treatment in the intensive care unit (mean difference = 1.47, 95% CI: -1.04, 3.96, *P* = 0.25) and the length of hospital stay (mean difference = 0.55, 95% CI: -3.90, 4.99, *P* = 0.81).

**Conclusion:**

The use of glucocorticoids may increase the mortality, the incidence of hospital-acquired pneumonia, and the need for mechanical ventilation in patients with severe pneumonia.

## 1. Introduction

Pneumonia is an infection of the lung that inflames the alveoli with resultant inflammatory secretions that prevent adequate oxygenation [1, 2]. During the infectious phase of pneumonia, excessive release of circulating inflammatory factors such as interleukin- (IL-) 10, IL-8, and IL-6 can lead to respiratory dysfunction [3]. An earlier study found that elevated levels of inflammatory factors increased patient mortality, especially in those with severe pneumonia that were associated with increased incidence of sepsis, lung injury, and acute respiratory distress syndrome (ARDS) [4]. Therefore, active and effective anti-inflammatory treatment is of great significance for severe pneumonia. Although severe pneumonia only accounts for about 10% of all pneumonia cases, it causes disproportionately high mortality [5]. Despite the continuous progress in antibiotic treatment and life support in recent years, the mortality associated with severe pneumonia has not decreased [5, 6].

Currently, glucocorticoid is the most effective anti-inflammatory medication. The therapeutic effect of glucocorticoids may be related to their ability to reduce the production of cytokines that mediate the inflammatory factor storm associated with severe pneumonia [7]. In addition, with the concept of critical illness-related corticosteroid insufficiency (CIRCI), glucocorticoid replacement therapy is gradually accepted in the field of critical medicine for conditions like sepsis and ARDS. Salluh et al. found that most patients with severe pneumonia suffered from adrenal crisis [8]. Some studies have also found that the low adrenaline level in the early stage of severe pneumonia was significantly correlated with unfavorable prognosis in severe pneumonia [9]. So far, many clinicians have used glucocorticoids in the treatment of patients with severe pneumonia, despite the optimal dose and administration frequency remain unclear.

Recent studies have shown that glucocorticoids may not improve the clinical outcome and may even increase mortality for severe pneumonia [10]. By contrast, many randomized controlled trials (RCT) have found that the use of glucocorticoids reduced the use of mechanical ventilation and the occurrence of ARDS in patients with severe pneumonia, shortened length of hospital stay, and reduced the 30-day mortality by 9% [11–13]. Therefore, there is still significant uncertainty regarding whether glucocorticoids can improve the prognosis of patients with severe pneumonia. Systematic meta-analysis can produce more reliable clinical evidence by combining the risk estimates of independent studies. Therefore, this study meta-analyzes the results from various RCTs to explore the role of glucocorticoids in improving the clinical outcome of severe pneumonia.

## 2. Methods

### 2.1. Bibliography Retrieval

This study used MeSH search words in PubMed, EMBASE, ScienceDirect, and other databases for literature retrieval. The search keywords are (“Pneumonia” [MeSH Terms] OR “acute respiratory distress syndrome” OR “acute respiratory failure”) AND (“Steroid, corticosteroid” [MeSH Terms] OR “glucocorticoid”) AND (“mortality” OR “hospital stay” OR “mechanical ventilation” OR “hospital acquired pneumonia” OR “ICU length of Stay”).

### 2.2. Literature Screening

Inclusion criteria: (1) the type of study design was RCT; (2) the study population was patients with confirmed severe pneumonia (PaO_2_/FiO_2_ < 300 mmHg); (3) the treatment method studied was glucocorticoid (not limited to a particular drug type, dosage, and duration). The control group was treated with placebo; (4) the primary endpoint included at least one of the following six categories: mortality, the incidence of mechanical ventilation, the incidence of secondary infection in the hospital, the length of hospital stay, length of treatment in intensive care unit, and length of treatment with mechanical ventilation.

Exclusion criteria: (1) the study population was limited to a special population, such as people with immune function defects or a special patient group; (2) reports with study population overlap; (3) the sample size of the interventional group or the control group was less than 20; (4) nonoriginal articles, such as discussions, academic conferences, reviews, and case reports; (5) studies with Newcastle-Ottawa Scale (NOS) score less than 5. This study did not limit the pathogens causing severe pneumonia and the age of patients.

### 2.3. Document Data Sorting and Evaluation

The two researchers screened and extracted the following data from the included literature independently: study type (open trial or double-blind trial), country or region of the study population, number of people in the control group and the interventional group, type of glucocorticoid use, mortality, the incidence of mechanical ventilation, the incidence of secondary nosocomial infection, length of hospital stay, length of intensive care unit treatment, and length of mechanical ventilation. This study used the Cochrane risk of bias tool for systematic reviews and meta-analyses of RCTs by two investigators independently to assess risk of bias for each included study based on seven aspects: (1) method of generating random numbers (selection bias), (2) group concealment (selection bias), (3) blinding of investigators and subjects (implementation bias), (4) blinding (detection bias) to the primary endpoint measure, (5) integrity of research results and data, (6) selective reporting, and (7) other biases. The evaluation criteria are as follows: (1) if the evaluation criteria are met, the risk of bias is low; (2) a risk of bias was considered possible if one or more of the criteria were only partially met or were less accurate; (3) a high risk of bias was considered to exist if one or more of the criteria were not met or not reported.

### 2.4. Statistical Method

STATA 17.0 (SE) was used in this study for the statistical analysis. The observed primary clinical endpoint was expressed by relative risk (RR) or mean ± standard deviation for categorical variables and continuous variables, respectively. Interstudy heterogeneity was assessed using the Cochrane *Q* test and the *I*^2^ statistic. For *I*^2^ ≥ 50%, the random effect model of the restricted maximum likelihood probability method is used to combine the mean difference and the RR. Otherwise, the fixed effect model of the reverse variance method is used. Meta-analyses with 5 or more included studies were evaluated for publication bias by funnel plot description and the Egger and Begg tests. All statistical results in this study were considered statistically significant at *P* ≤ 0.05, and the hypothesis tests were two-sided.

## 3. Results

### 3.1. Search Results and Literature Characteristics

A total of 382 relevant literature were generated. Regarding the established literature inclusion criteria, a total of 12 studies [13–24] were finally included in the meta-analysis. The detailed literature retrieval and screening process is shown in the flowchart (Figure 1). The characteristics of the 12 included papers are shown in Table 1. A total of 8171 patients were included in these 12 studies, with 12 reported mortality-related indicators, 7 reported length of stay indicators and ICU length of stay, 6 evaluated secondary nosocomial infection caused by glucocorticoid use, and 10 reported the number of patients using mechanical ventilation and the time of mechanical ventilation in the interventional and control groups. Six studies used two or more types of glucocorticoids, including methylprednisolone, dexamethasone, prednisolone, and hydrocortisone. It was found that 3 literature did not describe the grouping concealment and blind method of randomized grouping that was considered to have a moderate risk of bias; the rest of the included studies were of mild risk of bias. The NOS score ranged from 5 to 8, including 9 high-quality documents, 3 medium-quality documents, and 0 low-quality documents.

### 3.2. Glucocorticoid-Related Mortality

A total of 8171 patients in 12 studies were pooled for assessing glucocorticoid-related mortality. The random-effect model was applied to combine the RR given the heterogeneity test indicated moderate heterogeneity (*H*^2^ = 3.21, *I*^2^ = 68.84%, *P* = 0.01). The meta-analysis results (Figure 2) showed that compared with the control group, the use of glucocorticoids significantly increased the risk of death in patients with severe pneumonia (RR = 1.44, 95% CI: 1.13, 1.84, *P* < 0.001). The funnel chart (Figure 3) showed absence of obvious publication bias.

### 3.3. Incidence of Glucocorticoid-Related Nosocomial Infections

Six studies with a total of 4767 patients were included. The heterogeneity test results were *H*^2^ = 5.43, *I*^2^ = 81.57%, and *P* < 0.001, so the random-effect model was used to combine the RR. Compared with the control group, the use of glucocorticoids significantly increased the risk of nosocomial infection in patients with severe pneumonia (RR = 1.36, 95% CI: 1.01, 1.82, *P* = 0.04, Figure 4). The funnel chart (Figure 5) indicated no obvious publication bias.

### 3.4. Incidence of Glucocorticoid-Related Mechanical Ventilation

The RR were pooled from 6 studies with a total of 4767 patients using the random-effect model given the high interstudy heterogeneity (*H*^2^ = 8.32, *I*^2^ = 87.98%, *P* < 0.001). The meta-analysis results (Figure 6) showed that compared with the control group, the use of glucocorticoids significantly increased the risk of mechanical ventilation in patients with severe pneumonia (RR = 1.62, 95% CI: 1.30, 2.02, *P* < 0.001). Obvious publication bias was noted (Figure 7).

### 3.5. Length of Hospital Stay

A total of 1000 patients in 7 studies were included in this study. After confirming high interstudy heterogeneity (*H*^2^ = 20.91, *I*^2^ = 95.22, *P* < 0.001), the random-effect model was used to combine the mean difference. The meta-analysis results (Figure 8) showed that compared with the control group, the use of glucocorticoids did not seem to significantly increase the length of hospitalization (mean difference = 0.55, 95% CI: -3.90, 4.99, *P* = 0.81). The funnel chart (Figure 9) showed obvious publication bias.

### 3.6. Length of ICU Stay

The results of the meta-analysis that combined a total of 2653 patients in 7 studies using the random-effect model (*H*^2^ = 3.15, *I*^2^ = 68.24%, *P* = 0.01) showed the use of glucocorticoids significantly increased the number of patients with severe pneumonia treated in the intensive care unit for about 1.47 days (mean difference = 1.47, 95% CI: -1.02, 3.96), and the difference was not statistically significant, *P* = 0.25, as shown in Figure 10. There was no obvious publication bias (Figure 11).

### 3.7. Duration of Mechanical Ventilation

A total of 730 patients from four studies were included in this study. The heterogeneity test results were *H*^2^ = 3.91, *I*^2^ = 74.45%, and *P* = 0.01, indicating moderate heterogeneity. The random-effect model was used to combine the mean difference. The meta-analysis results (Figure 12) showed glucocorticoids did not significantly reduce the need for mechanical ventilation maintenance treatment in patients with severe pneumonia (mean difference = −1.10, 95% CI: -4.72, 2.51, *P* = 0.55). The funnel chart (Figure 13) showed no obvious publication bias, as shown in Figure 13.

## 4. Discussion

A total of 8171 patients with severe pneumonia were included in this study, including 1083 deaths. The all-cause mortality caused by severe pneumonia was 13.3%, which was comparable to that reported in the previous literature. In this study, 2301 patients needed mechanical ventilation. In addition, there were 1012 patients with secondary nosocomial infection. The main results of this study are as follows. (1) The use of glucocorticoids could increase the all-cause mortality of patients with severe pneumonia. (2) Glucocorticoid use increased the risk of requiring mechanical ventilation. (3) The incidence of nosocomial infection was higher in the glucocorticoid group than in the control group.

Usually, clinicians prefer to use glucocorticoids for adjuvant treatment in the early stage of severe pneumonia. The current clinical evidence supports the application of glucocorticoids in severe pneumonia for the following three reasons. First, glucocorticoids are potent inhibitors for the stimulation of the inflammatory cascade induced by pathogenic infection. Some studies proposed that the occurrence of the majority of severe pneumonia was usually related to excessive and uncontrolled inflammatory response. However, the exact anti-inflammatory mechanisms of glucocorticoids has not been fully clarified (3). However, it has been demonstrated that glucocorticoids play an essential role in activating genes that can encode anti-inflammatory factors and inhibit the expression of proinflammatory cytokines [25, 26]. In a case report of mechanical ventilation complicated with *Pseudomonas aeruginosa* infection, antibiotics combined with glucocorticoids has been shown to effectively reduce the inflammatory response, reduce the burden of bacterial proliferation in lung tissue, and improve the histopathological changes of the lung caused by inflammation [27]. In addition, critical illness-related corticosteroid insufficiency, which has been associated with excessive inflammation, was noted in 0-48% of patients with severe pneumonia. Moreover, some studies have found that the level of glucocorticoids could reasonably predict the severity of pneumonia [28].

On the other hand, it has also been known that glucocorticoids may exert a negative effect in patients with severe pneumonia with its associated immunosuppressive effect. Many pathogenic bacteria in hospital-acquired pneumonia are drug-resistant bacteria, such as *Clostridium difficile*, *Pseudomonas aeruginosa*, and *Acinetobacter baumannii*. A prior study that assessed the clearance of virus in vivo by real-time polymerase chain reaction reported slower virus clearance in the high-dose glucocorticoid group as compared with other groups [29]. Another study corroborated that slower virus clearance was associated with higher mortality in patients with ARDS [30].

This meta-analysis incorporated RCTs that were of high-quality and the research subjects covered a wide range of patient population, rendering the research conclusions potentially generalizable. In the meantime, this study also suffered from several limitations. (1) The sample size of a small part of the literature included in this study is relatively small, compromising statistical power and accuracy. (2) There are certain differences in terms of the definition of severe pneumonia among studies. Due to the differences with regard to patient characteristics, physician subjective judgment, and the various scoring scales used, it is difficult to reach a unified standard for the diagnostic criteria. These different characteristics may have a certain impact on the outcome of severe pneumonia treated with glucocorticoid. Therefore, the clinical diagnosis of severe pneumonia should be as comprehensive as possible, including demographic characteristics, clinical characteristics, imaging findings, laboratory examinations, and etiological tests. (3) The best scheme (including dose and administration frequency) for glucocorticoids in patients with severe pneumonia has not been fully clarified in the clinical guidelines. Previous studies have found that the type and dosage of glucocorticoids and glucocorticoid titering will have a certain impact on the clinical outcome. Due to the significant differences in the administration schemes between studies, it is impossible to uniformly determine the type and frequency of glucocorticoids. Therefore, glucocorticosteroid type and dosage differences may account for the medium to a high degree of heterogeneity in some subgroup analyses in this study.

In conclusion, we noted that glucocorticoid use was associated with increased all-cause mortality, elevated incidence of hospital-acquired pneumonia, and the need for mechanical ventilation.

## Figures and Tables

**Figure 1:** PRISMA flowchart. The process of screening meta-analysis into the literature.

**Figure 2:** Forest diagram of the effect of glucocorticoids on mortality of severe pneumonia.

**Figure 3:** Funnel diagram of the effect of glucocorticoids on mortality of severe pneumonia.

**Figure 4:** Forest chart of the effect of glucocorticoids on the incidence of hospital-acquired pneumonia in severe pneumonia.

**Figure 5:** Funnel chart of the effect of glucocorticoids on the incidence of hospital-acquired pneumonia in severe pneumonia.

**Figure 6:** Forest diagram of the effect of glucocorticoids on the incidence of mechanical ventilation in severe pneumonia.

**Figure 7:** Funnel diagram of the effect of glucocorticoids on the incidence of mechanical ventilation in severe pneumonia.

**Figure 8:** Forest diagram of the effect of glucocorticoid on the length of hospitalization of patients with severe pneumonia.

**Figure 9:** Funnel diagram of the effect of glucocorticoid on the length of hospitalization of patients with severe pneumonia.

**Figure 10:** Forest diagram of the effect of glucocorticoids on the length of time patients with severe pneumonia need to be treated in the intensive care unit.

**Figure 11:** Funnel diagram of the effect of glucocorticoids on the length of time patients with severe pneumonia need to be treated in the intensive care unit.

**Figure 12:** Forest diagram of the effect of glucocorticoids on the duration of mechanical ventilation in patients with severe pneumonia.

**Figure 13:** Funnel diagram of the effect of glucocorticoids on the duration of mechanical ventilation in patients with severe pneumonia.

**Table 1:** Characteristics of 12 included literatures.

Author	Study design	Location	Setting	Intervention/placebo	Corticosteroids used	Mortality outcome (12)	Length of hospital stay (d) (7)	Length of ICU stay (d) (7)	ARDS incidence	Nosocomial infection (6)	Mechanical ventilation required (d) (mean ± SD) (10, 4)
Tongyoo et al. [14]	RCT	Thailand	In hospital	98/99	50 mg hydrocortisone intravenously every 6 h daily/normal saline on the same time schedule	22/27 RR 0.82 (0.5-1.34)	NA	NA	22/27	17/19	16 ± 9.7/18.3 ± 10/ 33/21
Ceccato et al. [24]	Post hoc analysis of RCT	Spain	ICU	56/50	Methylprednisolone	2/1 HR 0.72 (0.11-5.44)	15.9 ± 17.3/16.4 ± 21.4	8.6 ± 11.4/7.9 ± 9.7	NA	NA	6/5
Nafae et al. [16]	Open-label RCT	Egypt	ICU	60/20	Hydrocortisone	4/6	9.27 ± 2.4/16.5 ± 2.24	3.1 ± 4.9/6.3 ± 8.2	NA	NA	8/5 1.2 ± 3.75/4.3 ± 7.83
Torres et al. [13]	Double-blinded RCT	Spain	In hospital	55/57	Methylprednisolone	6/9	11 (7.5-14)/ 10.5 (8-15) 11 ± 17.5/10.5 ± 18.9	5 (3-8)/6 (4-8) 5 ± 13.5/6 ± 10.8	NA	NA	5/10
Wittermans et al. [21]	Double-blinded RCT	Netherlands	In hospital	203/198	Dexamethasone	4/7	4.5 (4-5)/5.0 (4.6–5.4) 4.5 ± 5.1/5.0 ± 4.1	NA	NA	NA	NA
Fernández-Serrano et al. [15]	Double-blinded RCT	Spain	In hospital	28/28	Methylprednisolone	0/1	10 (9-13)/12 (9-18) 10 ± 7.64/12 ± 17.2	6.5 (5.5-9)/10.5 (6.25-24.5) 6.5 ± 6.68/10.5 ± 33.8	1/2	NA	1/5
Moreno et al. [17]	Propensity score matching study of RCT	Spain	ICU	604/1242	Methylprednisolone, prednisolone, or dexamethasone	166/234	NA	10 (5–19)/8 (5–18) 10 ± 23.1/8 ± 24.1	NA	139/248	506/921
Li et al. [18]	RCT	China	In hospital	1055/1086	Hydrocortisone, methylprednisolone, or dexamethasone	261/76	NA	NA	NA	227/154	367/49
Lee et al. [19]	RCT	Singapore	In hospital	612/2037	Hydrocortisone, methylprednisolone, or dexamethasone	70/33 HR 1.7 (1.1-2.6)	NA	NA	NA	NA	NA
Kim et al. [20]	Open-label RCT	Korea	ICU	107/138	Methylprednisolone or dexamethasone	62/37	30.8 ± 36.9/18.9 ± 20.0	13.5 ± 13.2/8.8 ± 9.2	66/70	61/30	91/71 13.3 ± 13.2/9.6 ± 10.0
Cao et al. [22]	Open-label RCT	China	In hospital	65/65	Hydrocortisone, methylprednisolone, or dexamethasone	27/10	NA	NA	NA	17/18	38/27
Brun-Buisson et al. [23]	Open-label RCT	France	ICU	83/125	Hydrocortisone, methylprednisolone, or hydrocortisone	28/21	23.2 (12.2-28.8)/18.1 (12.1-29.8)	22 (13–39)/17 (11–30)	NA	38/44	76/56 10.2 (9.8-16.8)/14.4 (13.2-23.3)

## Data Availability

The data used to support the findings of this study are included within the article.
